The article "Risk Factors for Unhealthy Weight Gain and Obesity among Children with Autism Spectrum Disorder" was published in 2019. Journal: Int J Mol Sci.

# Risk Factors for Unhealthy Weight Gain and Obesity among Children with Autism Spectrum Disorder

**DOI:** 10.3390/ijms20133285

**Published:** 2019-07-04

**Authors:** Khushmol K. Dhaliwal, Camila E. Orsso, Caroline Richard, Andrea M. Haqq, Lonnie Zwaigenbaum

**Affiliations:** 1 Department of Pediatrics, Faculty of Medicine and Dentistry, University of Alberta, 11405 87 Avenue, Edmonton, AB T6G 1C9, Canada; 2 Department of Agricultural, Food and Nutritional Science, Faculty of Agricultural, Life & Environmental Sciences, University of Alberta, 2-06 Agriculture Forestry Centre, Edmonton, AB T6G 2P5, Canada

**Keywords:** Autism spectrum disorder, ASD, Obesity, Overweight, Body mass index, BMI

## Abstract

Autism Spectrum Disorder (ASD) is a developmental disorder characterized by social and communication deficits and repetitive behaviors. Children with ASD are also at a higher risk for developing overweight or obesity than children with typical development (TD). Childhood obesity has been associated with adverse health outcomes, including insulin resistance, diabetes, heart disease, and certain cancers. Importantly some key factors that play a mediating role in these higher rates of obesity include lifestyle factors and biological influences, as well as secondary comorbidities and medications. This review summarizes current knowledge about behavioral and lifestyle factors that could contribute to unhealthy weight gain in children with ASD, as well as the current state of knowledge of emerging risk factors such as the possible influence of sleep problems, the gut microbiome, endocrine influences and maternal metabolic disorders. We also discuss some of the clinical implications of these risk factors and areas for future research.

## 1. Introduction

Autism Spectrum Disorder (ASD) is a developmental disorder characterized by social and communication impairments and repetitive behaviors [1,2]; the global prevalence is estimated at 1 in 160 children [3], although current North American estimates are around 1 in 60 children [4,5]. Children with ASD are also often at an increased risk for becoming obese (i.e., body mass index [BMI]-for-age ≥95th percentile) or overweight (i.e., BMI-for-age ≥85th percentile) than children with typical development (TD) [6,7,8]. These BMI levels are associated with adverse health outcomes, including insulin resistance, diabetes, heart disease, and certain cancers [9,10]. Obesity in childhood can also adversely affect physical, emotional, and social functioning, as well as academic performance [11], which might compound disability and reduced quality of life associated with ASD.

Some known key factors that may play a mediating role in the higher rates of obesity observed in children with ASD include eating behaviors [12], lifestyle [13], secondary comorbidities [14], and medications usage [15]. There is also evidence showing that reduced gut microbiota diversity [16,17], hormonal imbalances [18,19,20], and maternal metabolic disorders [21,22] may influence the development of either ASD or childhood obesity alone. However, it is yet not clear whether and to what extent these emerging factors are contributors for unhealthy weight gain and obesity among children with ASD. We define emerging risk factors as factors independently associated with increased risk for both obesity and ASD that have not yet been studied as risk factors for unhealthy weight gain and obesity among children with ASD.

Preventing unhealthy weight gain and obesity among children with ASD is crucial, as obesity affects overall children’s health and well-being and often persists into adulthood [23]. To develop appropriate strategies with increased efficacy, a comprehensive understanding of the risk factors for obesity development in ASD is required. Therefore, the purpose of this narrative review is to critically summarize current knowledge of behavioral, lifestyle, and biological factors potentially contributing to unhealthy weight gain in children with ASD. We also discuss the current state of knowledge of novel emerging risk factors for pediatric obesity in ASD.

Briefly, studies discussed in this manuscript were obtained after conducting a literature search in the main databases MEDLINE, CINAHL, and Google Scholar from inception to May 2019. We searched for multiple variations of the disorder (e.g., autism, autism spectrum disorder, Asperger syndrome) and keywords related to each section of this manuscript (e.g., obesity, overweight, weight gain, oral sensitivities, food selectivity, physical activity, recreational activities). Search was limited to articles in English and reference lists of selected articles, systematic reviews, and meta-analyses were manually reviewed to identify additional relevant articles. A critical synthesis of the literature is presented throughout the main text, describing the limitations of included articles.

## 2. Feeding Behavior

Reported rates of atypical behavior related to sensory experiences are high among children with ASD [24]. Compared to sex- and age-matched controls, individuals with autism aged 3 to 56 years old exhibited an abnormal oral sensory processing, characterized by either greater oral seeking (e.g., child putting everything into their mouth) or oral defensiveness (e.g., avoidance of certain textures and tastes and/or only eating a limited variety of foods) [25,26]. Interestingly, age-group analyses revealed reductions in the differences of sensory processing difficulties between ASD and TD children over time, suggesting that children are the most affected ones [25]. These sensory difficulties can lead to atypical eating behaviors and feeding practices in ASD, as children may avoid certain foods due to texture and/or taste and only eat a limited variety of foods (i.e., food selectivity). In fact, a recent meta-analysis identified that children with ASD experienced about five times more feeding problems and exhibited lower intake of calcium than TD children [27]. Thus, children with ASD may be at risk for inadequate micronutrient intake [28].

Although several studies characterizing feeding behaviors in children with ASD have evaluated the prevalence of overweight and obesity, few have attempted to investigate whether differences in feeding behavior are related to body weight categories. To our knowledge, only one study found that male children with ASD, who were overweight or obese, had more problematic mealtime and feeding behaviors than overweight or obese TD children, as indicated by the higher scores on a Behavior Pediatrics Feeding Assessment Scale (BPFA) in the ASD group [29]. There were no differences in BPFA scores between children with ASD and TD children, of either thin or adequate weight status [29]. However, another study of younger male and female children described no differences in feeding behaviors (assessed by questionnaire depicting oral function, eating problems, and others) across weight categories [30]. It is important to note that the sample populations in these two studies differed by age, sex, and cultural origins (Brazilian vs. Chinese), limiting comparison. Moreover, the second study found that children with ASD actually had lower mean BMI z-scores than TD children. Another approach to assessing whether feeding behaviors play a role in obesity is to examine within sample correlations. For example, one study found no significant association between dietary patterns and BMI z-score in children with ASD aged 3 to 11 years [31]. Therefore, it is not clear from the current literature whether feeding behavior is, and to what degree, a contributor to excess weight gain in children and adolescents with ASD. We speculate that abnormal feeding behaviors and/or dietary intake could influence weight status. For example, a study found children with ASD tended to consume more sweetened beverages and snacks foods (chips, candy, etc.) [31]. Thus, although children may be eating a limited variety of foods, these may be unhealthier overall (driving weight gain). However, picky eating could also result in weight loss [32].

Overall total energy intake and macronutrient distribution could also contribute to weight gain among children with ASD. With regard to total energy intake, two recent meta-analyses included three-day food record and food frequency questionnaires (FFQs) data from six prospective studies [27] and 14 observational studies [27,33]. No significant overall differences in total energy intake were detected between children with ASD and TD children [33]. It is also important to consider macronutrient distribution, which can lead to variations in body weight and cardiometabolic risk profiles [34,35]. However, the optimal macronutrient distribution for improving the weight status of children and adolescents is not yet understood [36]. Data from the same two meta-analyses that examined energy intake also assessed macronutrient intake, finding no significant difference in the intake of carbohydrates and fats between children with ASD and TD children [27,33]. Intake also tended to be within the acceptable macronutrient distribution range (AMDR) [8,33]. Children with ASD consumed less protein than TD children [27,33], but both groups were consuming more protein than currently recommended for a healthy diet [33].

Micronutrients are also integral to maintaining healthy body weight and have important functions in various metabolic pathways [37]. Children with ASD are often placed on restrictive diets, such as the gluten-free, casein-free (GFCF) diet [38], which may reduce intake of certain micronutrients. GFCF diets have been considered as a possible therapeutic intervention for some of the behavioral symptoms of ASD; however, evidence is lacking [39]. A recent systematic review identified three studies showing that nutrient inadequacies tended to remain among children with ASD even after controlling for common elimination diets, such as GFCF regimens [27,40,41,42]. Evidence suggests that deficiencies of vitamin A, vitamin D, B-complex vitamins, calcium, and zinc may be associated with increased fat deposition [43]. Findings from a meta-analysis confirm intake deficiencies in calcium and vitamin D in children with ASD relative to TD children and dietary intake recommendations [33]. However, the causality in the relationship between micronutrient intake and fat deposition remains unestablished [43]. Future studies should also take into account the use of dietary supplements, which are commonly offered to children with ASD [39].

In addition to these feeding behaviors and patterns, anecdotal reports indicate that children with ASD may limit their intake of fruits and vegetables due to factors such as taste and texture [42]. The consumption of fruits and vegetables has shown to be inversely associated with weight change and body adiposity [44,45]. However, studies based on prospective three-day food records generally demonstrate no difference in the intake of vegetables or fruits between children with ASD and TD children [40,46], with both groups consuming below the recommendations for vegetable intake [46]. In contrast, a systematic review of studies using FFQs (which assess subjective, longer-term eating patterns) indicated that children with ASD consume fewer daily servings of fruits and vegetables [31]. Likewise, Bandini et al. found that FFQ data revealed children with ASD refuse more vegetables than TD children [42]. In agreement with this, a study found that food refusal in children with ASD may in some cases be due to a bitter taste sensitivity associated with the TAS2R38 genotype [47]. Although little research has investigated the implications of polymorphisms in taste receptors and feeding behaviors in ASD, previous research has demonstrated that TD children exhibit two sensitive alleles for bitter taste had a lower threshold concentration to detected sucrose and a greater sugar consumption compared to children with less sensitive alleles [48]. Thus, future research into the prevalence of genetic variants of taste receptors in ASD may help to provide further insight into particular eating behavior differences, such as vegetable intake, among groups [49].

Overall, much of the recent literature seems to suggest that among those with ASD, overall intake of energy and macronutrients is fairly comparable to the TD population. These findings, however, must be interpreted with caution, because methods for collecting dietary information are often limited by variances in day-to-day food intake [50], under-reporting of energy intake [51], and behavioral reactions to measurement (e.g., changes in food intake, especially in individuals with obesity) [52]. Furthermore, although FFQs are designed to capture long-term eating habits, they include a limited number of foods and both FFQs and three-day food recalls are prone to recall bias [53]. Thus, the relationship between dietary intake and obesity rates may be clouded by limitations in these commonly used measures. In addition, parents of children with ASD may be more attuned to their children’s food selectivity behaviors, than parents of TD children, influencing diet data collection. Future studies using direct methods, such as doubly labeled water, to measure energy expenditure and energy intake, may be more informative [52,54]. Additionally, researchers should further elucidate differences in dietary intake within the ASD group based on oral sensitivities, dietary restrictions, and secondary comorbidities (e.g., GI disorders), and take into account age- and possibly sex-related differences. Eating disorders, such as anorexia nervosa, can also impact feeding behaviors and studies have found comorbidities between eating disorders and ASD, specifically among females [55,56]. Studies suggest that specific behavioral phenotypes, such as rigid and repetitive behaviors and social anhedonia, overlap among both conditions [56,57]. This further highlights the importance of stratifying feeding behaviors based on sex differences.

## 3. Physical Activity and Sedentary Behavior

School-based or extracurricular programs provide opportunities for children to be physically active and engage with peers. Physical activity (PA) is considered a protective factor in maintaining a healthy body weight and preventing obesity [58]. However, opportunities for PA may be limited in children with ASD due to social and behavioral challenges [59,60], as well as motor deficits [61,62,63].

For optimal health benefits [64], the U.S. Department of Health and Human Services Office of Disease Prevention and Health Promotion suggests that children between the ages of 6 and 17 years should engage in moderate- to vigorous-intensity physical activity (MVPA) for at least 60 min, 3 days per week [65]. Studies that have assessed intensity and frequency of PA in children and adolescents with ASD are summarized in Table 1. Studies comparing the daily time spent in MVPA, as measured by accelerometers, between children with and without ASD have yielded mixed findings. For example, while Bandini et al. reported similar daily MVPA in children with ASD and TD children [66], Stanish et al. found that children with ASD who are younger than 16 years old spent less time engaged in MVPA; but for those adolescents over 16 years, the difference in MVPA was not significant [67]. In contrast, a systematic review found a consistently negative association between PA and age [68]. The discrepancies in these findings suggest that longitudinal studies would enhance the understanding on whether age influences PA patterns. Notably, both children with ASD [67] and TD children [69] were unlikely to meet the recommendations for MVPA.

Studies utilizing parent report questionnaires generally show that children with ASD spend less time engaged in PA than TD children [70,71,72]. Although questionnaires are more feasible than objective measures given the associated time demands and costs, parent-reports often underestimate PA [73]. In the Bandini et al. study, parents reported that their children with ASD spent significantly less time in PA annually (158 vs. 225 h per year) and participated in fewer types of PA, but no differences in PA between children with ASD and TD children were observed based on accelerometry data [66]. Parents of children with ASD also report more barriers to PA (e.g., increased needs for supervision), which could influence their estimates of overall PA [70]. Moreover, a weak to moderate correlation has been found between parent reports of children’s PA and accelerometer-measured activity, depending on type of activity and age group [73]. It is possible that children react to being monitored by increasing their PA [74]; on the other hand, social desirability bias could cause parents to under- or over-report their children’s PA based on weight status [75].

Another important variable to consider is sedentary behavior (SB), which is defined as resting behavior with very little expenditure of energy [76]. Factors contributing to prolonged SB in children may include increased access to television, computers, and phones [77,78]. Prolonged SB has long-term health consequences, such as increased body weight, cardiovascular diseases, and type 2 diabetes [79,80]. In a recent systematic review, only two of six studies comparing the prevalence rates of SB reported greater participation in SB by children with ASD than TD children [68]. However, children with ASD (aged 8–18 years old) spent 62% more time on screen activities compared to their TD siblings, as reported by parents [81]. Furthermore, children with ASD spent more hours per day playing video games (both boys and girls), but spent less time using social media or playing interactive video games [81,82].

Overall, the relationships between time spent in MVPA or SB and the propensity for children with ASD to be overweight or obese were not directly investigated in the reviewed studies. It is important to note that ASD severity may influence these relationships by affecting behavior as well as social and motor functioning [83]. Indeed, McCoy et al. found an association between higher parent-reported levels of autism severity, increased odds of being obese, and decreased odds of PA [71]. In the future, research based on objective measures of MVPA and SB (e.g., accelerometer data) could yield insights into differences in these variables between children with ASD and TD children. Further sample stratification based on ASD severity could further clarify how symptoms moderate the relationship between PA and SB among children with ASD.

## 4. Genetics

Genetic vulnerabilities and syndromic causes of ASD and obesity have been explored extensively, albeit independently. Both conditions are heritable; thus, understanding possible shared genetic links may yield insights into their interplay. Specifically, sibling and twin studies have shown that ASD tends to run in families [84,85]. Likewise, genetics also play a role in childhood obesity [86]. When compared to adopted siblings, the risk of being obese is higher among individuals with affected siblings and parents who are already obese [87]. Because both ASD and obesity have heritable components, investigation of any genetic overlap in their pathways may help explain the higher rates of obesity among individuals with ASD.

Sharma et al. hypothesized that a common molecular pathway may contribute to the pathogenesis of ASD and obesity, as a pathway-based analysis revealed 36 common genes between these two conditions [88]. Specifically, one study has shown that ASD, Attention Deficit Hyperactivity Disorder (ADHD), developmental delays and obesity are highly associated with a microdeletion involving 11p14.1 [89]. Furthermore, deletions in 16p11.2 were associated with genetic vulnerabilities related to both obesity and ASD [90,91]. More recently, in a genetic analysis of very obese children with ASD, Cortes and Wevrick focused on de novo mutations and found that very obese ASD probands had loss of function mutations in DNMT3A and POGZ [92].

In addition, Prader-Willi Syndrome (PWS) is a genetic disorder caused by paternal 15q11–13 deletions [93]. PWS is characterized by hyperphagia, elevated ghrelin concentrations, and increased risk for obesity [93,94]. PWS is also associated with higher rates of social-communication impairments and repetitive behaviors [95], although the degree to which symptoms meet diagnostic criteria for ASD varies across studies, emphasizing that ASD symptom measures require careful consideration of developmental profile and overall clinical context [95,96]. That said, genetic mechanisms underlying the association between Prader Willi and ASD may underlie obesity risk related to hyperphagia in a subset of individuals with ASD [97].

In summary, although evidence indicates that certain genetic vulnerabilities are associated with both ASD and obesity, there is a need to further investigation, such as pathway-based analyses to reveal how genetics influence the complex etiologies of both conditions. In addition, it is not currently clear what proportion of children with ASD and obesity would be accounted for by these rare genetic variants; future efforts to parse the relative contribution of genetic versus non-genetic associations would provide important insights into this topic. Genetic testing, in the form of clinical microarrays, are increasingly becoming standard of practice for ASD diagnosis [98] and determining whether there are deletions in areas such as 16p11.2 may allow for early interventions and targeted molecular therapy, with potential to prevent obesity in children with ASD.

## 5. Medications

Comorbid conditions, such as ADHD and depression, often manifest in ASD [99]. To manage these and other behavioral symptoms, psychotropics including stimulants, selective serotonin reuptake inhibitors (SSRIs), and antipsychotics are often prescribed [100]. The prescription rate of these drugs in children with ASD has been reported at 27–64% (median 41.9%) [101,102,103,104].

A 2016 meta-analysis by Park found that 1 in 6 children with ASD were prescribed anti-psychotic medication [105]. Second-generation anti-psychotics (SGA) such as risperidone and aripiprazole, are often prescribed to alleviate behavioral symptoms comorbid with ASD such as hyperactivity, irritability and aggression [106,107], but are associated with substantial weight gain [15,106]. A systematic review of seven randomized controlled trials (RCTs) of risperidone use among children and adolescents with ASD, revealed weight gain as an adverse event [15]. Furthermore, dose-related increases in blood glucose, insulin, and leptin have been reported [108] and metabolic changes (e.g., leptin) track closely with changes in fat mass [109]. Furthermore, a systematic review looking at two RCTs of apriprazole use in children with ASD reported a mean difference of 1.13 kg of weight gain in children using apriprazole compared to a placebo after 8 weeks of treatment [110]. Other commonly prescribed antipsychotics in ASD are olanzapine and clozapine [111,112]. A 2014 meta-analysis found that olanzapine and clozapine were also both associated with severe weight gain [113]. The mechanism of action behind weight gain associated with atypical antipsychotics relates in part to serotonin receptor blockade and reduction in dopamine (D2) receptor-mediated neurotransmission [114], implicated in weight regulation [115]. Thus, monitoring adverse effects of antipsychotics are important to alleviate behavioral symptoms without detrimental effects on metabolic health [116].

Selective serotonin reuptake inhibitors (SSRIs) are another class of medications commonly prescribed to children with ASD for comorbid anxiety, depression and obsessive-compulsive behaviors [117,118]. Previous research on the efficacy of citalopram [119] and fluoxetine [120] in children with ASD have not examined changes in weight gain. However, other research has suggested SSRIs such as citalopram may cause weight gain [121]. The degree and persistence of weight gain with these medications, particularly from long term use, are not known in children with ASD, and thus would benefit from further study.

## 6. Emerging Factors

### 6.1. Breastfeeding

Breast milk provides energy, nutrients and antibodies, and reduces risks for various infections during infancy [122]. Researchers have also studied how breastfeeding affects children’s cognitive development. The rate and duration of exclusive breastfeeding also appears to be a potential risk factor for ASD [123]. For example, Boucher et al. found associations between longer durations of breastfeeding and better cognitive development and fewer autistic traits in children, after controlling for relevant demographic and social confounding variables [124]. Tseng et al. also reported that children with ASD were significantly less likely to have been breastfed than children without ASD [123]. Tseng et al. highlighted some proposed explanations for the role of breastfeeding in ASD pathophysiology, such as the nutrition theory [125], oxytocin stimulation [126], and the secretion of neurotrophic factors [123,127].

Researchers have also found that breastfeeding may lower the risk of childhood obesity [128,129]. In their meta-analysis, Yan et al. showed a dose-response effect between breastfeeding duration and reduced risk of childhood obesity [130]. These studies highlight that reduced breastfeeding may be a contributing factor to obesity, although they did not specifically examine these relationships in ASD. Thus, future studies could examine how breastfeeding affects the growth patterns and long-term weight status of children with ASD.

### 6.2. Sleep

Evidence suggests that sleep duration and quality of sleep are risk factors for becoming overweight or obese [131]. Numerous studies have confirmed an inverse correlation between sleep quantity, BMI, and the risk for overweight and obesity [132,133]. A 2016 meta-analysis found an association between poor sleep quality (independent of sleep duration) and overweight and obesity in children [134]. Decreased quality of sleep can lead to endocrine changes affecting appetite regulation and glucose metabolism, with implications on body weight gain [135]. As such, an inverse relationship between total sleep and ghrelin levels has been reported, as well as a positive relationship between total sleep and leptin levels [136]. Ghrelin and leptin are appetite regulating hormones that influence food intake. Childhood obesity can present with sleeping problems such as obstructive sleep apnea (OSA) [137]. OSA is associated with inadequate duration and poorer quality of sleep and may be associated with specific metabolic markers such as insulin resistance and hypertension [137].

Studies have found that children with ASD have higher rates of sleep problems when compared to TD controls [138]. One study found associations between poor sleep quality and weight status among children with ASD, with 86% of the obese group presenting with clinically significant sleep problems compared to 76% of those with healthy weight [139]. Children with ASD are more likely to be diagnosed with insomnia, circadian rhythm disorder, or sleep-disordered breathing such as OSA [140]. Metabolic risk factors, as well as day-time sleepiness, may reduce daytime activity levels, contributing to unhealthy weight gain [139]. Although many findings suggest that children with ASD are at greater risk for sleep problems, associations with BMI remain underexplored within this population. However, sleep duration and quality are important factors to consider, because increased findings of sleep problems may be compounding the risk for unhealthy weight gain in children with ASD.

### 6.3. Microbiota

Gastrointestinal (GI) disorders, such as diarrhea, chronic constipation [141], and abdominal pain are common in ASD [142]. In a study including 163 preschoolers with ASD, 25.8% of the participants reported having at least one severe GI symptom [143]. Studies have also shown that children with ASD and GI problems have higher levels of affective problems, including anxiety, than children with ASD who have normal GI functioning [14,143,144]. This link between GI and behavior disorders suggests that gut microbiota may influence developmental course in ASD [145].

Data from several pediatric studies reveals a unique gut microbiota profile in children with ASD compared to those with TD, but inconsistent findings on the characterization of the bacterial communities [146]. While one study reported decreased bacteria of the genera *Prevotella*, *Coprococcus* and *Veillonellaceae*, other studies found increased *Lactobacillus*, *Clostridium*, *Candida* spp., and the Firmicutes/Bacteroidetes ratio [16,146,147,148]. Similar to what has been seen in ASD, studies exploring the gut microbiome in obesity have reported an increased Firmicutes/Bacteroidetes ratio, and this ratio could be positively associated with BMI in children and adults with obesity [149,150,151]. To further understand the implications of obesity on gut composition, animal studies comparing lean, wild-type, and obese mice (leptin-deficient) have demonstrated an increase in the Firmicutes/Bacteroidetes ratio in obese mice, independent of diet [152]. Indeed, a high-fat diet was shown to promote more profound increases in Firmicutes [153]. Certain features of the gut microbiota, such as individual variability, may explain the lack of a consistent microbiota signature in ASD and obesity. As the gut microbiota is assembled mainly during infancy, before the age of 2 years, diverse factors including birth mode, antibiotics, feeding practices, and environmental exposure to bacteria shape the gut community and contribute to this individual variability [154]. Thus, characterizing the microbiome from an ecological perspective (bacterial diversity, abundance, community interactions, metabolic profiles), may be more informative in understanding the interplay between gut microbiota, ASD prognosis, and weight gain.

Growing evidence suggests that decreased gut microbiota diversity in ASD [16,155] may be associated with behavioral and GI symptoms. Sharon et al. took this hypothesis a step forward, reporting that offspring of germ-free mice receiving gut microbiota from individuals with ASD indeed exhibited behaviors related to those observed in ASD [156]. This finding, however, must be interpreted with caution given the small sample size used in the experiments and relevance to behavioral expression in the human condition.

Gut microbiome dysbiosis, which refers to changes in the composition and function of gut microbiome especially early in life, are associated with increased production of pro-inflammatory cytokines and alterations in the dynamics of the communication between the gut and brain, known as the gut-brain axis [157,158,159]. These cytokines affect the inflammation pathways, which have been implicated in ASD development [158,159,160]. Inflammatory cytokines and an increased gut permeability also promote metabolic endotoxemia [161], which plays a role in the development of obesity and metabolic diseases [162]. Indeed, gut microbiome dysbiosis has also been reported in obesity [163].

A much-debated topic is whether gut permeability contributes to ASD development [159], with evidence remaining limited and controversial. To our knowledge, only three studies have investigated gut permeability in children with ASD using varied biomarkers [164,165,166]. Specifically, children with ASD exhibited greater gut permeability than TD children, as assessed by zonulin concentrations [164] or sugar probes (lactulose and mannitol) [165]. In contrast, no difference in gut permeability using the lactulose and rhamnose probe was observed in children with ASD compared to TD children [166]. There were marked differences in the design of these studies; in particular, with respect to the selection of comparison groups. One study included children with and without GI complaints in both study (i.e., children with ASD) and control (i.e., children with TD) groups; another study excluded children with GI symptoms from the control group only; and in the third study, all children (study and control groups) had mild GI disorders. Thus, it is not clear whether gut permeability is increased due to the presence of ASD or GI-associated disorders per se. Furthermore, studies have shown significantly lower short-chain fatty acids (SCFAs) in ASD [167]. As SCFAs are produced by gut microbiota (from dietary fiber fermentation), and their production promotes gut barrier and mucosal integrity [168], it could be speculated that individuals with ASD may have decreased ability to repair the intestinal barrier.

Dietary intake has a direct impact not only on obesity development, but also on the microbiome composition [169]; the role of diets in ASD could thereby be explored as a possible way to alleviate both irritable bowel syndrome symptoms and some ASD problem behaviors. An interesting avenue to explore would be fiber interventions in ASD, especially in those children with concomitant obesity. Many studies have found that fiber intake in children with ASD, as well as TD, does not meet recommended levels [8,42]. Fiber-rich foods can alleviate GI symptoms, such as chronic constipation and increase feelings of fullness, as these foods take longer to digest [170]. Fiber intake could also promote a healthier metabolic profile by mediating the gut microbiota [171,172]. Our bodies produce SCFAs by degrading fiber in the gut, which results in the release of anorexigenic gut hormones [173], improvements of the gut barrier [174], and triggering of anti-inflammatory cytokines [175,176]. More specifically, the SCFA propionate was shown to promote increases in peptide YY (PYY) and glucagon like peptide-1 (GLP-1) levels in an in vitro study using human colonic cells [177]. Subsequent in vivo studies were conducted in human adults; while acute intake of inulin-propionate ester reduced energy intake by ≈14% with increases in plasma PYY and GLP-1, supplementation over 24 weeks reduced rate of weight gain and intra-abdominal adiposity [177]. In addition to alleviating GI symptoms associated with ASD, SCFAs thus also prevented obesity and its comorbidities [178]. However, sensory aversions (e.g., to food texture) associated with ASD may create challenges with increasing intake of fiber rich foods.

Further delineating the microbial signature of individuals with comorbid ASD and obesity may provide further insight into the complex etiologies of both conditions. Although more studies are needed, there is emerging evidence of a dysbiotic gut microbiome influencing children with ASD. If supported by more definitive studies (e.g., metagenomics), evaluation of novel therapeutic strategies would be warranted, such as dietary interventions and fecal transplantations. Some challenges in this area include the need for approaches to directly sample the gut mucosa in order to reliably characterize the microbiome in various group and regions [179]. Furthermore, animal studies remain difficult to translate because of the precise control over genetics, the environment, and diet; which is not possible in human studies, making the human microbiome a lot more heterogeneous [179].

### 6.4. Endocrine Influences

Researchers have also begun to explore the role of endocrine factors in the pathogenesis of ASD. It has been hypothesized that specific chemical messengers, such as endocrine hormones, and neuropeptides work together with neurotransmitters (e.g., dopamine and serotonin) to influence the developing fetal brain [20]. Thus, imbalances in the chemical transmissions could lead to defective encoding, which could in turn lead to some of the social behaviors exhibited by those with ASD [20]. Research in this area has been focused on understanding how hormonal imbalances and differences may contribute to the pathogenesis of ASD. In this section, we review evidence related to specific appetite hormones, leptin, adiponectin and ghrelin.

### 6.5. Leptin

Leptin is an anorexigenic (satiety) hormone that regulates how much one consumes and inhibits appetite [180]. Produced by adipose tissue in amounts proportionate to fat mass [181], leptin is an important hormone involved in energy homeostasis and growth [182]. Evidence suggests that obese individuals exhibit leptin resistance, whereby the brain no longer responds to leptin by inhibiting energy intake and increasing energy expenditure [183,184].

Several studies have reported higher circulating concentrations of leptin in individuals with ASD compared to control groups [18,19,185,186,187,188], summarized in Table 2. Ashwood et al. found higher concentrations of peripheral blood leptin in individuals with ASD compared to age-matched controls, despite no group differences in BMI [18]. Leptin plays an important role in growth [182] and rapid growth has also been independently implicated as a risk factor for ASD [189]. One study found that children born small-for-gestational age (SGA) had lower leptin cord levels; among those born SGA, children with the most rapid weight gain had the highest childhood leptin levels and were more likely to be diagnosed with ASD [187], suggesting differences in early weight trajectories between children with ASD and TD children [7]. Hasan et al. measured fasting serum concentrations for 20 children with ASD and 20 TD children; the BMI of the group with ASD was significantly lower compared to the control group; however, no children in either group were found to be of obese status [188]. The study found that the children with ASD had higher leptin concentrations and lower BMI [188], suggesting that leptin concentrations could be higher among individuals with ASD, regardless of weight status. The studies summarized in Table 2 have consistently found higher concentrations of leptin in children with ASD when compared to TD children. In the future, leptin concentrations could be analyzed based on BMI percentile stratifications to explore relationship to obesity among children with ASD.

### 6.6. Adiponectin

Adiponectin is a protein hormone secreted by the adipocytes [190]. Plasma adiponectin levels and BMI are strongly negatively correlated in both men and women [191]. Adiponectin is an anti-inflammatory protein [192]; decreased levels may lead to increased expression of adhesion molecules and inflammatory molecules, resulting in higher risk for cardiovascular diseases associated with obesity [193]. Therefore, adiponectin and its receptors may be therapeutic targets for individuals who are obese or overweight [193,194].

Disturbances in immunoinflammatory factors and adipocytokines have been reported among individuals with ASD relative to age- and weight-matched TD controls [195]. Table 3 summarizes published data on adiponectin concentrations in children with ASD compared to controls [19,186,196,197]. One study reported lower serum adiponectin levels among individuals with ASD relative to age- and sex-matched healthy controls [196], but two other studies showed no significant differences [19,186]. Differences in findings among the three studies may be explained by differences in exclusion and inclusion criteria and sample composition, particularly by sex and age. For example, Rodrigues et al. and Blardi et al. included both males and females, whereas Fujita-Shimizu et al. only included males [19,186,196]. Past studies have found sex differences in adiponectin levels and body composition [198,199], whereby adiponectin concentrations decrease into late puberty and become significantly lower in males by adulthood [199]. Furthermore, recent findings also suggest a link between a high leptin/adiponectin ratio (i.e., higher concentrations of leptin and lower concentrations of adiponectin) and abdominal obesity [200]. Although higher concentrations of leptin among individuals with ASD is a relatively consistent finding, the role of adiponectin is less clear. Exploring the relationship between these two hormones and its potential role in the propensity for individuals with ASD to become overweight or obese warrants further examination.

### 6.7. Ghrelin

Ghrelin is an appetite-stimulating hormone [201], but its exact role in obesity is poorly understood, as, counterintuitively, ghrelin is often suppressed in obese individuals, and concentrations increase with weight loss [202]. Evidence about the role of this hunger hormone in children with ASD is also unclear. Researchers have explored serum ghrelin concentrations in two case control studies of children with ASD (see Table 4). One study found that male children with ASD had significantly lower concentrations of acylated, des-acylated, and total ghrelin [185]. However, findings from a more recent study, that included both boys and girls, showed a trend towards lower concentrations of ghrelin, although not significant, in children with ASD when compared to age-matched TD children [188]. Previous studies have found that ghrelin levels can be modified by an increase in sex hormone [203], whereby testosterone can lead to marked decreases in ghrelin [203], which may contribute to differences in findings between these two studies. Future studies should examine ghrelin levels relative to weight status as well as ASD diagnosis and consider sex differences.

Although researchers have begun to explore the role of hormones in contributing to higher rates of obesity among children with ASD, they have focused primarily on hormonal differences in relation to ASD pathogenesis. Furthermore, some of the studies discussed above did not report a difference in BMI or weight status among children with ASD, when compared to TD children. However, the relatively smaller sample sizes, compared to larger scale studies (which have reported greater rates of obesity in children with ASD), may have contributed to these differences in findings [6,7]. Future studies, which stratify study groups based on weight status (overweight, obese, etc.), sex, and age would help to understand whether there are potential biological differences associated with specific weight status. Therefore, further research into possible differences in these hormones’ concentrations, in children with ASD, may yield insights into hormonal impacts on unhealthy weight gain and obesity.

### 6.8. Maternal Metabolic Disorders

Although maternal metabolic disorders such as diabetes, hypertension and obesity could place children with ASD at higher risk for becoming overweight or obese, this hypothesis has not been explored directly. Instead, researchers have focused on examining maternal metabolic disorders as potential risk factors for ASD in children; separately, others have studied how maternal metabolic disorders may increase risk of obesity in children.

Maternal obesity prior to pregnancy is a risk factor for ASD [21,204,205]. Evidence has also shown significant associations between maternal diabetes and hypertension and ASD risk [206,207,208]. Several mechanisms may contribute to these in-utero effects. In a systematic review, Xu et al. suggested several potential pathways through which maternal diabetes may increase the risk for ASD in offspring: (a) maternal hyperglycemia can result in hypoxia and impair neural development in the fetus [209,210,211] (b) maternal hyperglycemia can cause oxidative stress associated with ASD risk [212,213], and (c) increased maternal adiposity can cause chronic inflammation that can affect neuronal development [206,214].

Concurrently, there has been considerable research on how maternal metabolic disorders may increase children’s obesity risk. In their systematic review, Wang et al. found a strong positive association between parental and child obesity and overweight status across various countries, indicating a genetic predisposition toward obesity, with other factors playing a mediating role, such as obesogenic lifestyles and behaviors [22]. In another recent systematic review and meta-analysis, Kawasaki et al. reported an association between gestational diabetes mellitus and higher BMI z-scores among offspring [215]. Deierlein et al. found an association between fetal exposure to maternal glucose concentration in the high–normal range and children being overweight or obese at 3 years of age, independent of maternal pre-pregnancy BMI [216]. Furthermore, Lawlor et al. conducted a sibling analysis to control for shared genetics and environment and reported that children exposed to diabetes in utero had higher BMI than their unexposed siblings [217].

These findings may help explain how certain maternal metabolic disorders increase risk for obesity. Factors such as lifestyle behaviors and genetic predisposition may have compounded effects on weight gain for children with ASD. Additional research on in-utero effects of maternal metabolic disorders may help explain why many children with ASD tend to become overweight or obese. Longitudinal studies to assess parental weight status and track neurodevelopmental outcomes and weight in offspring would provide important insights into the extent to which parental obesity status influences the development of obesity in children with ASD. A better conceptualization of the role of maternal metabolic disorders and any shared pathophysiology between ASD and obesity would help mothers understand how to best reduce their children’s risk for both health conditions.

## 7. Future Directions and Perspectives

The current treatments for childhood obesity generally involve a combination of (1) non-pharmacological interventions (e.g., behavioral treatments, weight-reducing diets), (2) pharmacological interventions, (3) and surgical treatments [23]. Typically, behavioral treatments and weight-reducing diets, such as family-based interventions, are the first therapeutic steps [218]. However, these may be problematic for children with ASD, who struggle with social and behavioral communication, changes in routine, and sensory processing difficulties [24,68]. Furthermore, challenges with self-management and, in many cases, impairments in decision-making skills play an important role in the challenges associated with this first line of treatment in children with ASD [219]. The second line of intervention is through common pharmacological treatments for childhood obesity, such as orlistat, sibutramine, and metformin. These, however, may cause abdominal pain, fecal incontinence, nausea, and vomiting [220,221]. Administering medications that can cause GI problems to children with ASD, who typically already have co-morbid GI disorders, may cause additional difficulties [222]. Moreover, because many children already take medication to manage symptoms of ASD and other comorbid medical conditions, additional medications may increase the risk of side effects, as well as pharmacological interactions and medication burden [223,224]. Finally, severe and morbid forms of pediatric obesity may warrant surgical interventions such as bariatric surgery [225]. Although the prevalence of severe morbid obesity (that would warrant consideration of bariatric surgery) among children with ASD is unclear, a study reported that children with the de novo 16p11.2 deletion, which is associated with autism, were also severely obese (BMI ≥ 120% of 95th percentile) [226]. Bariatric surgery, however, also comes with its risks and complications associated with Roux-en-Y gastric bypass, such as pulmonary embolism, shock, intestinal obstruction, postoperative bleeding, staple line leaks and severe malnutrition [23]. Furthermore, adolescents are more likely to have remission of type 2 diabetes and hypertension after bariatric surgery, when compared to adults [227], emphasizing that optimal timing for surgery in order to reverse metabolic complications of obesity is still unclear. Furthermore, little research has been done in this area to address treatment needs that may be specific to this population [219]. A systematic review looking more broadly at children with intellectual disabilities suggested the need for further research into how obesity treatment can be more specifically tailored for children with intellectual disabilities [219]. Finding more intensive treatments and combination of techniques are warranted for children with intellectual disabilities, such as more training for parents to support children with defiant behaviors [219,228].

Furthermore, although much is known about behavioral and lifestyle factors, little is known about possible biological drivers of obesity among children with ASD. There is also a need to identify whether specific biological drivers can be monitored and assessed at an earlier age, such as at the time of ASD diagnosis. Research in this area is particularly important, because evidence suggests that weight trajectories, at an earlier age, may be different among children with ASD. Therefore, clinical health surveillance of these weight trajectories in ASD and monitoring of growth patterns may serve as a useful method in preventing unhealthy weight gain and obesity. Based on this review, biological factors (gut microbiota, endocrine hormones, maternal metabolic disorders) may be driving increased propensity to become overweight, but further research is needed. Finally, given some of the unique challenges faced by children with ASD, results from pediatric obesity trials in the general population may not generalize to patients with ASD. Thus, as a field, we may require more targeted treatment options and ASD-specific randomized, controlled trials. In an era of precision medicine, there is a need to take into account the interplay between behavioral and biological characteristics influencing unhealthy weight gain in ASD.

## 8. Conclusion and Recommendations

Body weight is determined by energy balance, which is influenced by environmental (e.g., nutrition), behavioral (e.g., food selectivity, PA, SB), and biological (e.g., genetics, metabolic dysfunction) factors. Because the etiologies of ASD and obesity are so complex, risk factors specifically associated with one condition or the other are difficult to disentangle. Nevertheless, it is important to understand that many risk factors for becoming obese or overweight are heightened in individuals with ASD, as suggested by growing evidence. Figure 1 summarizes the risk factors discussed within this review. A limitation of this narrative review is that we compared various risk factors for unhealthy weight gain and obesity in children with ASD to TD children. Although similarities were found with regard to specific risk factors between children with ASD and TD children (i.e., physical activity, etc.), this does not necessarily mean these are not clinically relevant to children with ASD and should still be taken into account in future studies, including clinical trials.

Overall, evidence suggests that oral sensitivities may mediate food selectivity and food and nutrient intake and other factor such as PA, SB, sleep, genetics, and medication usage may all contribute to some degree, and ultimately have a compounded effect on weight gain in ASD. Additionally, researchers have begun to investigate the roles of sleep problems, the gut microbiome, the endocrine system, and developmental risk factors. Going forward, studies of obesity in ASD should incorporate assessment of both biological and lifestyle-related factors, as well as test for mediating and moderating relationships such as ASD severity, oral sensitivities, and sex and age differences. It is important to consider these multiple factors in conjunction with individual factors to clarify whether unhealthy weight gain affects children across the entire ASD spectrum, or whether certain children are more vulnerable than others. Understanding each of these individual risk factors and components is important to effectively prevent and treat unhealthy weight gain among children with ASD and to facilitate the development of potential early intervention strategies. An understanding of individual risk factors would enable the development of personalized approaches to help children with ASD manage their weight, including dietary recommendations, medical therapies, and nutrition and exercise regimens. Overall in conjunction with the clinical guidelines for pediatric obesity [229] and ASD care [98], clinicians should consider more tailored medical surveillance in children with ASD that considers the above factors in a care and management plan.

## Figures and Tables

**Figure 1:** Risk factors for becoming obese or overweight among individuals with ASD. Primary factors include risk factors which have been directly implicated in obesity and/or unhealthy weight gain, in children with ASD. Secondary factors are those which are not specific to children with ASD but could result in unhealthy weight gain. Emerging factors are those on which we have postulated hypotheses based on indirect evidence. *Created with BioRender.

**Table 1:** Physical activity.

Study	Design	Study Group	Control Group	Measure	Result	BMI
Bandini et al. [66]	Cross-sectional	53 male and female children with ASD (age: 3–11 years)	58 male and female TD children (age: 3–11 years)	Accelerometer data Questionnaire (parent report on type and frequency)	Similar daily MVPA for both groups (ASD: 50.0 min/day; TD: 57.1 min/day). Children with ASD participate in significantly fewer types of physical activities (6.9 vs. 9.6, *p* < 0.0001) and spend less time annually participating in these activities than TD children (158 vs. 225 h per year, *p* < 0.0001).	No significant difference between the two groups BMI-z score not significantly associated with percent time spent in MVPA
Stanish et al. [67]	Cross-sectional	35 male and female children with ASD (age: 13–21 years)	60 male and female TD children (age: 13–18 years)	Accelerometer data (total average daily PA) Questionnaire (type and frequency of PA)	Children with ASD who are younger than 16 spend less time in MVPA (ASD: 26 min/day vs. 51 min/day) and participate in fewer activities. No significant difference in MVPA among individuals older than 16 years.	N/A
Must et al. [70]	Cross-sectional	53 children with ASD (age: 3–11 years)	58 TD children (age: 3–11 years)	Parent report questionnaire (type and frequency)	An inverse correlation between the total number of barriers reported and the number of PA hours per year (ASD: 119 h; TD 169 h; *p* < 0.05).	No significant difference in BMI percentiles
McCoy et al. [71]	Cross-sectional	915 male and female children with ASD (age: 10–17 years)	41,879 male and female TD children from the 2011–2012 National Survey of Children’s Health (age: 10–17 years)	Parent report questionnaire (type and frequency)	Adolescents with ASD are less likely to engage in PA (*p*< 0.05) Higher autism severity is associated with increased odds of being obese (OR: 2.8; 95% CI: 1.39, 3.74), and decreased odds of PA (OR: 0.30; 95% CI: 0.20, 0.46).	Adolescents with ASD are more likely to be overweight and obese (ASD: 22%; TD 14.1%; *p*< 0.05).
Healy et al. [72]	Cross-sectional	67 male and female children with ASD (age: 13 years)	74 randomly selected male and female TD children (age: 13 years)	Parent report questionnaire (type and frequency)	Significantly lower participation in MVPA (*p* < 0.001) and sports reported for children with ASD (*p* < 0.001).	No statistically significant difference between the two groups in mean BMI and overweight/obese status.

**Abbreviations:** ASD, Autism Spectrum Disorder; TD, Typically Developing; MVPA, Medium–Vigorous Physical Activity; BMI, Body Mass Index.

**Table 2:** Leptin in ASD.

Study	Design	Study Group	Control Group	Measure	Result	BMI
Ashwood et al. [18]	Case control	70 male and female children with ASD (age: 2–15 years)	50 age matched TD children	Peripheral plasma concentrations of leptin	Leptin levels were higher in children with autism compared with typically developing non-ASD controls (*p* < 0.006)	No statistical differences in BMI or z-scores between ASD or controls
Blardi et al. [19]	Case control	35 male and female children with ASD (mean age 14.1 years)	35 TD sex and age matched children	Baseline: 6 mL blood sample after an overnight fast 1 year after: 6 mL blood sample after an overnight fast	Leptin concentrations of children with ASD were significantly higher than TD children at baseline (*p* < 0.001) and after a year *(p* < 0.001)	No significant difference between children with ASD and TD children on weight or height at baseline or after 1 year BMI z-score not provided
Al-Zaid et al. [185]	Case control	31 male children with ASD (age: 3–8 years)	28 age- and sex-matched TD children (age: 3–8 years)	7 mL of venous blood samples were collected after an overnight fast	Leptin concentrations were higher in the group with ASD when compared to the TD group (*p* ≤ 0.01)	Weight was higher in the children with ASD (19.3 kg in TD children and to 22.7 kg in children with ASD) (*p* = 0.05) No significant difference in BMI between groups (*p* = 0.28)
Rodrigues et al. [186]	Case control	30 male and female children with ASD (ages not provided)	19 TD children matched for age, gender, maternal age at child birth	10 mL plasma blood samples	Plasma levels of leptin were higher (*p* < 0.01) in children with ASD, compared to TD children	Article suggests differences in BMI (unclear of significance and values)
Raghavan et al. [187]	Prospective cohort	39 male and female children with ASD	616 male and female TD children	Plasma umbilical cord blood sample and non-fasting childhood (median age= 18.4 months) venous blood sample	Mean cord leptin was lower in children later diagnosed with ASD (*p* = 0.05) Children with the highest leptin levels had an increased ASD risk (OR: 5.41; 95% CI: 1.53, 19.05)	Birthweight was greater in TD children and compared to children with ASD (*p* = 0.03) Extremely rapid weight gain was associated with greater ASD risk
Hasan et al. [188]	Case control	20 children with ASD (16 males and 4 females) (mean age: 5.9 years)	20 age matched TD children (13 males and 7 females) (mean age: 6.0 years)	5 mL blood samples from participants (serum)	Serum levels of leptin were higher in children with ASD compared to TD children (*p* = 0.038)	TD children had greater mean weight (*p* < 0.001), height (*p* < 0.001), and BMI (*p* < 0.05), compared to children with ASD

**Abbreviations:** ASD, Autism Spectrum Disorder; TD, Typically Developing; BMI, Body Mass Index

**Table 3:** Adiponectin in ASD.

Study	Design	Study Group	Control Group	Measure	Result	BMI
Blardi et al. [19]	Case control	35 male and female children with ASD (mean age 14.1 years)	35 TD sex and age matched children	Baseline: 6 mL blood sample after an overnight fast 1 year after: 6 mL blood sample after an overnight	Adiponectin levels in autistic patients were not significantly different from those found in controls at each time.	No significant difference between children with ASD and TD children on weight or height at baseline or after 1 year BMI z-score not provided
Fujita-Shimizu et al. [196]	Case-control	31 male children with ASD (age: 6–19 years)	31 age-matched male TD children (age: 6–19 years)	Fasting blood samples	Serum levels of adiponectin in the group with ASD were significantly lower (*p* = 0.005) than the TD group	No significant difference in weight, height, waist circumference, and BMI between the two groups BMI z-score or BMI weight categories not provided
Rodrigues et al. [186]	Case control	30 male and female children with ASD (ages not provided)	19 TD children matched for age, gender, maternal age at child birth	10 mL of blood (plasma)	No difference in the plasma concentration of adiponectin in children with ASD compared to TD children	Articles suggests differences in BMI (unclear of significance) BMI z-score or BMI weight categories not provided
Raghavan et al. [197]	Prospective cohort	55 male and female children with ASD	792 male and female TD children	Plasma umbilical cord blood sample and non-fasting childhood (median age = 19.03 months) venous blood sample	Mean cord blood adiponectin was higher in TD children compared to the group with ASD (*p* = 0.01) No significant difference in early childhood adiponectin	Birthweight was greater in TD children and compared to children with ASD (*p* = 0.03) Extremely rapid weight gain was associated with greater ASD risk

**Abbreviations:** ASD, Autism Spectrum Disorder; TD, Typically Developing; BMI, Body Mass Index.

**Table 4:** Ghrelin in ASD.

Study	Design	Study Group	Control Group	Measure	Result	BMI
Al-Zaid et al. [185]	Case control	31 male children with ASD (age: 3–8 years)	28 age- and sex-matched TD children (age: 3–8 years)	7 mL of venous blood samples were collected after an overnight fast	Acylated ghrelin concentrations were lower in the group with ASD than TD children (*p* ≤ 0.001) Deacylated ghrelin concentrations were lower in group with ASD compared to TD children (*p* ≤ 0.005)	Weight was higher in the children with ASD (19.3 kg in TD children and to 22.7 kg in children with ASD) (*p* = 0.05) No significant difference in BMI or height BMI z-score or BMI weight categories not provided
Hasan et al. [188]	Case control	20 male and female children with ASD (16 males and 4 females) (mean age: 5.9 years)	20 age-matched healthy control children (13 males and 7 females) (mean age: 6.0 years)	5 mL blood samples from participants (serum)	Serum levels of ghrelin were lower in children with ASD compared to TD children, but not statistically significant (*p* =0.32)	TD children had a greater mean weight (31.17 kg), height (1.32 m^2^), and BMI (17.6 kg/m^2^) compared to children with ASD with a mean weight of 21.26 kg, height of 1.17 m^2^, and BMI of 15.5 kg/m^2^ BMI z-score or BMI weight categories not provided

**Abbreviations:** ASD, Autism Spectrum Disorder; TD, Typically Developing; BMI, Body Mass Index.

## Abbreviations

ADHD	Attention Deficit Hyperactivity Disorder
AMDR	Acceptable Macronutrient Distribution Range
ASD	Autism Spectrum Disorder
BMI	Body Mass Index
BPFA	Behavior Pediatrics Feeding Assessment Scale
FFQ	Food Frequency Questionnaire
GFCF	Gluten-Free Casein-Free
GI	Gastrointestinal
GLP-1	Glucagon-Like Peptide- 1
MVPA	Moderate- to Vigorous-intensity Physical Activity
OSA	Obstructive Sleep Apnea
PA	Physical Activity
PYY	Peptide YY
PWS	Prader-Willi Syndrome
RCT	Randomized Controlled Trial
SB	Sedentary Behavior
SCFA	Short-Chain Fatty Acid
SGA	Second Generation Antipsychotic
SSRI	Selective Serotonin Reuptake Inhibitors
TD	Typically Developing
